This article has been retracted.

# Application Value of Remote ECG Monitoring in Early Diagnosis of PCI for Acute Myocardial Infarction

**DOI:** 10.1155/2022/8552358

**Published:** 2022-08-08

**Authors:** Jian Zhou, Jun Li

**Affiliations:** First People's Hospital of Chenzhou City (Emergency Department), Chenzhou, 423000 Hunan, China

## Abstract

The blockage of blood in the vessels results in heart attacks and cardiac arrests which are referred to as myocardial infarction. Early detection of such infarction is feasible through percutaneous coronary intervention (PCI) based on electrocardiogram (ECG) monitoring. The variations in blood flow and clot are precisely observed through periodic ECG monitoring and previous correlations. This article introduces a concentrated value assessment model (CVAM) for determining PCI levels in treating myocardial infarction. The ECG observations from the previous observation sessions are accumulated and organized for validating the infarction rate. This requires the accompanying concentrated data like a heartbeat, blood pressure, and flow rate observed in different sessions. Based on the session observation and normal data correlation, the PCI level is recommended for the patient. In this analysis process, the value shift due to blocks and high and low blood pressure is accounted for through the deep learning paradigm. This paradigm correlates the above factors with the ECG values for precisely determining PCI from the last known concentration. The learning paradigm is trained based on session and normal observation data through different intervals. This model is validated using the metrics precision, analysis rate, diagnosis recommendation, and complexity.

## 1. Introduction

Electrocardiography (ECG) placed an important role in healthcare applications because it is used to diagnose cardiovascular disease (CVD) [1]. The patient health status is continuously observed with the help of ECG monitoring [2]. Several literature analyses are frequently performed to improve the patient health status. However, the traditional research analysis handles several difficulties while diagnosing patient health reports. The developed system should support monitoring needs; from the reference of various literature analyses, the ECG monitoring system has been created according to the expert's idea [3]. In [4], numerous classification peer-studies are conducted to enhance the overall ECG monitoring efficiency. The study gives the ECG monitoring system characteristics, relationship, and challenges used to optimize ECG system performance. Therefore, a general architectural model of an ECG monitoring system is proposed, and a comprehensive analysis of the value chain of the ECG monitoring system is performed [5, 6]. Finally, key challenges were identified, and the importance of smart surveillance systems was highlighted, which utilizes artificial intelligence (AI), deep learning (DL), Internet of Things (IoT), and big data techniques widely utilized to create effective systems [7].

Ischemic heart disease (CHD) is a more crucial and severe death-related disease. CHD is treated with the help of a percutaneous coronary intervention (PCI) procedure. The PCI is one of the nonsurgical invasive processes created to rectify the obstructed coronary arteries and enhance ischemic tissue blood flow [7, 8]. The PCI procedures are widely applied in the coronary artery disease treatment process. Due to the importance of CHD in [9], the detailed percutaneous disease information is described along with the caretaking procedure [10]. During the treatment process, the radial artery or femoral is utilized for accessing the blood flow. Then, fluoroscopy is applied for visualizing the catheter and tissue position [11]. The advanced version of the ascending aorta is defined as a catheter that is presented in the coronary arteries. It has both left and right arteries. In the treatment process, contrast agents are applied to the coronary artery that has been viewed in the anatomy. The coronary artery images are taken from various angles and position that give detailed information about the disease [11, 12].

This disease is highly correlated with mortality; acute myocardial and morbidity infarction remains the main focus of cardiovascular disease management. In addition, data on 30-day acute myocardial infarction mortality and readmission rates are published to promote its awareness [13, 14]. Percutaneous coronary intervention remains an important treatment when the patient has coronary artery symptoms, especially acute myocardial infarction. It has received widespread attention over the past decade due to concerns such as the benefits and risk of combination therapy with antithrombotic therapy and drug-eluting stents received [15, 16]. This is especially important as the process of updating clinical guidelines and quality scores for acute myocardial infarction and percutaneous coronary intervention are accelerating However, few representative data are describing current treatment regimens and outcome trends in patients with acute myocardial infarction undergoing percutaneous coronary intervention [16, 17].

## 2. Related Works

Hussain and Park [18] introduced a cyberphysical cardiac monitoring system named Big ECG for stroke management. Wearable ECG sensors play a major role in collecting the information which is related to a patient's health condition and provide the necessary set of data for the monitoring process. Medical ontology and data analytics are used here to find out the defects and problems in the monitoring process which improves the accuracy rate in the detection process [19]. The proposed system improves the performance and feasibility of the system.

Bigler et al. [20] proposed a new intracoronary electrocardiogram (ECG) method for the myocardial ischemia detection process. ECG collects data via signals which provide necessary ECG parameters for the detection process. ECG parameters are reasonable and contain every detail about intracoronary details [21]. The proposed method increases the accuracy rate in the detection process which enhances the efficiency of the system.

Jiao et al. [22] introduced a capsule network-assisted electrocardiogram (ECG) classification model for smart healthcare systems. The defined model is mostly used for identifying the type of cardiovascular disease. The feature extraction process is done using a convolutional neural network (CNN) and long short-term memory (LSTM) algorithm which find out the optimal features [23]. The feature extraction process extracts both temporal and special features which are given by ECG signals. The proposed model provides an accurate set of data for further data analysis and detection processes in healthcare systems.

Tadesse et al. [24] introduced a deep multilead electrocardiogram (ECG) fusion method (DeepMI) for myocardial infarction (MI) detection in healthcare systems. ECG first collects data that are related to MI and produces a feasible set of data for the detection process. The fusion strategy is used here to find out the time occurrence of MI via signals. The proposed method reduces the latency rate in the classification process which improves the energy consumption rate in the computation process. The proposed DeepMI method increases the feasibility and efficiency of healthcare systems.

Zhao et al. [25] introduced an artificial intelligence- (AI-) based ST-segment elevated myocardial infarction (STEMI) detection method using an electrocardiogram (ECG). AI technique is used here to identify the accurate set of data for the detection and classification process. The proposed method is mostly used in healthcare applications to find out STEMI patients among others [26]. Experimental results show that the proposed method increases the accuracy rate in the detection process which improves the efficiency and scalability of the system.

Fatimah et al. [27] proposed a new myocardial infarction (MI) detection method using single-lead electrocardiogram (ECG) signals. The Fourier decomposition method (FDM) is used here to remove the baselines of MI features that are collected by ECG. The *K*-nearest neighbor (KNN) algorithm is also used in the proposed method to find out the difference among the data and produce an optimal set of data for the detection process [28]. The proposed MI detection method increases the overall accuracy rate in the detection process which provides better performance and feasibility of the system.

Han and Shi [29] proposed a novel myocardial infarction (MI) detection method using a multilead residual network (ML-ResNet). A single-lead feature branch network is used here to train the dataset which is required for the MI detection process. Both spatial and temporal features are extracted using the feature extraction process and produce an optimal set of data for the detection process. Experimental results show that the proposed ML-ResNet method achieves a high accuracy rate in the classification and location process which enhances the effectiveness of the system.

Li et al. [30] introduced a new automated myocardial infarction (MI) detection model (SLC-GAN) using a generative adversarial network for healthcare applications. A single-lead electrocardiogram (ECG) signal is used here which provides related data for the monitoring process via wearable devices. The proposed SLC-GAN method automatically finds out the MI by using a convolutional neural network (CNN). When compared with other methods, the proposed SLC-GAN method improves the accuracy rate in the MI detection process which increases the diagnosis process in healthcare applications.

Aldana Blanco et al. [31] introduced a new electrocardiogram (ECG) sonification method for myocardial infarction (MI) monitoring and diagnosis processes in healthcare systems. Polarity sonification is a parameter-mapping method that format synthesizer to get related information for the mapping process. The proposed method identifies the danger stages of patients which reduce the complexity rate in the MI diagnosis process. The proposed method increases the accuracy rate in the detection and classification process which reduces the latency rate in the diagnosis stage.

Thorén et al. [32] proposed a new electrocardiogram (ECG) monitoring process for in-hospital cardiac arrest (IHCA) in the healthcare system. The main purpose of the method is to identify the features and details of patients which provide a proper set of data for the monitoring process. The proposed method improves the propensity scores (PS) in the ECG monitoring process. The proposed method reduces the complexity rate in the diagnosing process by improving the accuracy rate in the MI classification and identification process.

Aldana Blanco [32] introduced a wearable electrocardiogram (ECG) signal monitoring method using the convolutional neural network (CNN) approach. ECG collects data from devices and produces an optimal set of data for the monitoring process. CNN is mainly used here for classification and data analysis processes which play a major role in the monitoring process. The spatial filtering method is used here to extract the features which are presented in collective ECG signals. The proposed method increases the overall accuracy rate in the classification and analysis process which improves the efficiency and effectiveness of the system.

Thorén et al. [32] proposed a new prediction method for the refusal of percutaneous coronary intervention in the myocardial infraction detection process. The proposed method identifies the patient's details that refuse the intervention procedure in healthcare application. The classification and regression tree (CART) analysis process is used here to find out the intervention details of the patients. The proposed method provides various sets of data for the detection and recognition process which improves the efficiency and feasibility of the system.

## 3. Proposed Concentrated Value Assessment Model

The design goal of CVAM is to monitor for early detection of myocardial infarction through PCI observation. The proposed ECG monitoring using PCI observation for heart attacks and cardiac arrest is designed to improve session observation, and data correlation of the PCI level is recommended for the patient. Early observation of such myocardial infarction through PCI observations based on ECG monitoring consecutively is for better heart attack detection for validating the infarction rate. The ECG observation requires the blood pressure, heartbeat, and flow rate observed in various sessions. In this process, the variations in blood flow and clot are computed through ECG monitoring, and a previous correlation is an important factor for which the analysis rate is to be thwarted through session and observation analysis. The CVAM makes use of a deep learning paradigm for the patient. In this proposed model, the ECG monitoring and PCI levels of the different session observations and previous correlations are considered to improve the analysis of PCI levels in treating myocardial infarction. From different session observations, the variations and complexity of the actual ECG observations from the previous observation sessions are unavailable.  Figure 1 presents the proposed model illustration.

The ECG data from different observation sessions are used for extracting the heartbeat, blood pressure, and flow rate concentrated values. This data is analyzed through deep learning for correlation. From this correlation process, variations (abnormality) and normal observations are identified (refer to Figure 1). The determining PCI level is based on periodic ECG monitoring and previous correlation used in treating cardiac arrest and heart attacks experiencing a different session observation that is to be monitored and analyzed for such infarction and early detection. This blockage of blood in the vessels of the patient is referred to as myocardial infarction in different sessions. In particular, ECG observations through the PCI level are prevented from complexities in different observation sequences to improve the diagnosis recommendation based on the infarction rate. However, to retain the variations in blood flow and clot from the human body observation, the proposed model provides session observation, and normal data correlation with high and low blood pressures are accounted for. The function of CVAM is to identify variations in blood flow and clot; the ECG observation from the patient is performed and is monitored between ECG monitoring and PCI observations. The treatment of myocardial infarction in early diagnosis through PCI value shift and heart rate is administered to prevent complexity in the above metrics with the ECG values for determining PCI levels from the last known concentration.

### 3.1. Problem Definition

Let {1, 2, ⋯, *p*} ∈ *P* denote the set of patient observations detected in different intervals *P*_*r*_ ∈ (*P*_*r*_^*M*^ − *P*_*r*_^*C*^), where *P*_*r*_^*M*^ and *P*_*r*_^*C*^ are the precision in ECG monitoring and previous correlation observations, respectively. Different analyses of PCI levels represent as PCI_*L*_, and the session observation *S*_ob_ must be less under observed instance based on treating myocardial infarction precision in various patient observation instances that are given by equations (1a) and (1b):

(1a) $$\begin{array}{c} \forall \left(P_{r}^{M}-P_{r}^{C}\right),\text{argmin }\overset{P_{r}}{\underset{t=1}{\sum }}{\left({\text{PCI}}_{L}-S_{\text{ob}}\right)}_{t},P_{r}\in \left[P_{r}^{M}+1,P_{r}^{C}\right]. \end{array}$$

Such that

(1b) $$\begin{array}{c} \text{argmin }\overset{S_{\text{ob}}}{\underset{t=1}{\sum }}{\left(C\right)}_{t},\forall \left\{1,2,\cdots ,p\right\}\in P,P_{r}^{M}\leq P_{r}\leq P_{r}^{C}. \end{array}$$

From equations (1a) and (1b), the variable *t* denotes the ECG monitoring time intervals and (PCI_*L*_ − *S*_ob_) is the session observation in different instances *P*_*r*_ ∈ [*P*_*r*_^*M*^ + 1, *P*_*r*_^*C*^]. This processing instance improves the previous correlation in different intervals, reducing the complexity of treating myocardial infarction.

The above issues are accounted for using the analysis precision and input patient observation of the real-time application value of remote ECG monitoring in early diagnosis of PCI for heart attacks and cardiac arrest through a deep learning paradigm. However, there are few conditions based on *P*_*r*_^*M*^ and *P*_*r*_^*C*^ that are computed as follows:

- ∀*p* ∈ *P* in [*P*_*r*_^*M*^, *P*_*r*_^*C*^], if the condition (*p* + 1) is true in *P*_*r*_ ∈ [*P*_*r*_^*M*^ + 1, *P*_*r*_^*C*^], then (*p* + 1) experiences previous observation sessions of (*P*_*r*_ + *P*_*r*_^*M*^ + 1), where *P*_*r*_ represents the blood pressure rate instances
- ∀*p* ∈ *P* in *P*_*r*_^*M*^, if *P*_*r*_ = *P*_*r*_^*C*^ or *P*_*r*_ > *P*_*r*_^*C*^, then the condition *C* = (PCI_*L*_ − *S*_ob_) is performed for ECG monitoring based on the condition PCI_*L*_/*S*_ob_⟶0

As per the conditions, variable *C* represents the complexity of identifying the blockage of blood in the vessels. The first condition represents the ECG observation instance of the (*P*_*r*_^*M*^ − *P*_*r*_^*C*^) where the next previous correlation is based on *p* heartbeat rate. Instead, the condition (*p* + 1) is analyzed with any *P*_*r*_ ∈ [*P*_*r*_^*M*^ + 1, *P*_*r*_^*C*^] of ob. This augments the precision and analysis rate for both *p* and (*p* + 1). Similarly, the second condition identifies the complexities and precision in identifying the variations in [*P*_*r*_^*M*^ − *P*_*r*_^*C*^] different intervals and also validating the infarction rate with the successive PCI_*L*_ provided argmin ∑_*t*=1_^*V*_*i*_^(*P*_*r*_^*M*^)_*t*_∀ [*P*_*r*_^*M*^ − *P*_*r*_^*C*^] is satisfied. The CVAM is administered based on the session observation and normal data correlation observed consecutively using the previous observation sessions. The ECG monitoring output and PCI level analysis for the patients in the real-time E-medical and E-healthcare application services rely on ECG values. The infarction rate (In_*r*_) of the patient input depends on the different sessions. However, the precision less application monitoring and observation are the concentrated value factor for In_*r*_. Hence, based on conditions (i) and (ii), In_*r*_ is computed as

(2) $$\begin{array}{c} {\text{In}}_{r}=\left(P_{r}^{M}+P_{r}^{C}\right)+\left(P_{r}^{M}-1+P_{r}\right)\forall P_{r}^{C}\leq P_{r}\leq P_{r}^{M}. \end{array}$$

The infarction rate factor must overlap with the precision and previous correlation analysis such that the condition *P*_*r*_ ∈ [*P*_*r*_^*M*^ + 1, *P*_*r*_^*C*^]∀ (*p* + 1) does not analyze complexity *P*_*r*_ ∈ [*P*_*r*_^*M*^, *P*_*r*_^*C*^]∀ *p* ∈ *S*_ob_. The above equation for In_*r*_ does not analyze ECG observations from the previous observation sessions as it differs in variations due to the analysis of blood flow and clots required in the human body. The early detection of myocardial infarction and session observation of the PCI level is observed based on *S*_ob_ that determines (PCI_*L*_ − *S*_ob_) and satisfies the condition PCI_*L*_/*S*_ob_⟶1. The value shift analysis due to blocks in the heart depends on In_*r*_ and [*P*_*r*_^*M*^, *P*_*r*_^*C*^]; those conditions are reduced by *C* of the previous session observation of the myocardial infarction. The above conditions (i) and (ii) are analyzed sequentially and identified heartbeat for both the ECR monitors and PCI level analysis of the applications using the deep learning paradigm. This deep learning helps to restore the previous observation sessions accumulated and organized for validating the optimal infarction output where finding precise myocardial infarction observation in previous correlation, precision, and analysis rate instance is achieved. Consecutively, the ECG observation-based infarction rate verification using deep learning is discussed. In Figure 2, *P*_*r*_^*C*^ and *S*_op_-based observation and classification process is illustrated.

The ECG data from different *S* ∈ OB is used for identifying CF_*D*_ and CF_*S*_. This  CF_*D*_ is identified from the current and previous correlation analysis whereas CF_*S*_ is the recent (current) observation. (PCI_*L*_, *P*_*r*_^*C*^) and (*S*_OP_, *P*_*r*_^*M*^ + 1) estimations are performed for identifying varying CF. This is further correlated using the neural process for shift (abnormality) detection. Based on this feature, the following cases are analyzed for session observation and last known concentrated values.

### 3.2. Condition (i) Analysis

This condition deals with the session observation and normal data correlation; the PCI level is recommended for the patient in previous observation required for analysis of blood pressure analysis in the successive data correlations. The first output for precisely determining PCI from the last known concentration is the diagnosis process in different intervals, and observation varies based on the ECG monitoring sequence of the blood pressure analysis of the session correlation. Initially, the data correlation of real-time applications based on the heartbeat and flow rate of the PCI_*L*_ relies on *P*_*r*_^*C*^ given as

(3) $$\begin{array}{c} \text{OB}\left({\text{PCI}}_{L},P_{r}^{C}\right)⟵\left(1-\frac{{\text{PCI}}_{L}}{P_{r}^{C}}\right)\frac{P_{r}}{P_{r}^{C}}+\frac{\left(P_{r}^{C}-P_{r}^{M}\right)}{\left(P_{r}^{C}+1\right)}\left[\arg\underset{S_{\text{ob}}}{\min}\frac{{\left(P_{r}^{C}\right)}_{\text{in}}}{{\left(P_{r}^{C}+1\right)}_{t+1}}\right]\forall t\in {\text{PCI}}_{L}. \end{array}$$

The above two observations (OB) based on the session and correlation can be extracted such that the condition OB(PCI_*L*_, *P*_*r*_^*C*^) is the rallying factor for the previous identification of myocardial infarction assessment instances for *P*_*r*_^*M*^ + 1 such that

(4) $$\begin{array}{c} \text{OB}\left(S_{\text{ob}},P_{r}^{M}+1\right)⟵\frac{{\text{In}}_{r}}{P-p}+\left(\frac{P_{r}^{M}+1}{P_{r}^{C}}\right)\left[{\left(P_{r}^{M}+1-P_{r}^{C}\right)}_{t}\right]\forall t\in S_{\text{ob}}. \end{array}$$

In the above equation (4), the second condition helps to construct the observation depending on *P*_*r*_^*C*^, *P*_*r*_^*M*^, and *P*_*r*_^*M*^ + 1 for a different instance of previous session observation, by monitoring the infarction rate for reducing complexities. The precise output is based on the analysis of session and normal observation data *P*_*r*_^*M*^ in different intervals. This analysis process is performed using deep learning. The deep learning process validates such infarction observed in different sessions, based on the condition OB(PCI_*L*_, *P*_*r*_^*C*^) and OB(*S*_ob_, *P*_*r*_^*M*^ + 1), respectively.  Figure 3 presents the learning representation for normal data correlation.

In Figure 3, the session-based normal data correlation is performed. In this correlation, the stored data is also utilized for identifying variations. The variation is observed if CF_*D*_ ∈ (*S* + 1) or (*D* + 1). Therefore, both inputs are utilized for training the neural network. In this neural network,∀*S*, *p* is mapped for (*S*_OP_, *P*_*r*_^*M*^) or (*S*_op_, *P*_*r*_^*M*^ + 1). This deep learning is performed for accounting the value shifts based on blocks and high and low blood pressure in the same interval *P*_*r*_^*C*^ ≤ *P*_*r*_ and *P*_*r*_^*C*^ ≤ *P*_*r*_ ≤ *P*_*r*_^*M*^ for preventing the severe complexity and diagnosis recommendation in session observation. As per the early detection of OB(*S*_ob_, *P*_*r*_^*M*^ + 1), the infarction is based on heart attack and cardiac arrest identification in the present patient observation *P*_*r*_ and thus requiring In_*r*_. However, this infarction rate does not overlap with the accumulated data sessions, and hence, the new session observation is determined. The new session observation instance admitting deep analysis for early detection of myocardial infarction must satisfy the condition *P*_*r*_^*C*^ ≤ *P*_*r*_ to prevent additional complexity metrics. Case (i) for either infarction rate as in equation (2) is processed, and blood pressure verification using the ECG values of OB(*S*_ob_, *P*_*r*_^*M*^ + 1) until *P*_*r*_^*C*^ ≤ *P*_*r*_^*M*^ the condition is satisfied. The concentrated value factor (CF) is computed for the condition *P*_*r*_^*C*^ ≤ *P*_*r*_ and *P*_*r*_^*C*^ ≤ *F*^*T*^ based on OB(PCI_*L*_, *P*_*r*_^*C*^) and OB(*S*_ob_, *P*_*r*_^*M*^ + 1) as in

(5) $$\begin{array}{c} {\text{CF}}_{D}=\left(1-\frac{{{\text{In}}_{r}}^{D}}{D}\right)+\left(\frac{{\left(P_{r}^{M}\right)}_{D}}{{\left(P_{r}^{C}\right)}_{D}}\right)-\left(\frac{{\left[C\right]}^{D-1}}{S_{ob}}\right),\text{for OB}\left({\text{PCI}}_{L},P_{r}^{C}\right), \end{array}$$

where

(6) $$\begin{array}{c} {\text{CF}}_{s}=\left(1-\frac{{\left[C\right]}^{s-1}}{s}\right)+\left(\frac{{\left(P_{r}^{M}\right)}_{s}-{\left(P_{r}^{C}\right)}_{s}}{P_{r}^{M}+S_{\text{ob}}+1-4\;}\right). \end{array}$$

The concentrated value factor correlates early detection *D* and sessions *s* observations in two instances; therefore, *P*_*r*_^*M*^ = *F*^*A*^ + 1  and ( *P*_*r*_^*M*^ + *S*_*o*_ + 1 − *P*_*r*_) = *P*_*r*_. In the final known concentration of CF_*s*_, if the condition *P*_*r*_^*M*^ + *S*_ob_ + 1 verifies the blood pressure continuously and the exceeding *p*, then the chances of complexity are detected. This *C* is addressed in computing case (ii).

In this deep learning, the conditions of *P*_*r*_ ≤ *P*_*r*_^*M*^, *P*_*r*_ ≤ *P*_*r*_^*M*^ + 1, and *P*_*r*_ < *P*_*r*_^*M*^ + 1 are to be achieved to satisfy the reliable output of PCI_*L*_. The session observation and normal data correlations based on myocardial infarction identification require heartbeat, blood pressure, and flow rate checking and interval verifications in PCI level observation. Therefore, the concentrated value factor for the above condition *P*_*r*_ ≤ *P*_*r*_^*M*^ and *P*_*r*_ ≤ *P*_*r*_^*M*^ + 1 are computed in a continuous manner of equations (5) and (6). This continuous process of value shift between the previous two intervals of ECG observations with the present instance is estimated as in equations (7) and (8):

(7) $$\begin{array}{c} {\text{CF}}_{s+1}=\left(1-\frac{P_{r}^{M}}{P_{r}^{C}+1\;}\right)+\left(\frac{{{\text{In}}_{r}}^{D}}{{\text{PCI}}_{L}-p}\right). \end{array}$$

Such that

(8) $$\begin{array}{c} {\text{CF}}_{D+1}=\left(1-\frac{{\left[C\right]}^{{\text{PCI}}_{L}}}{S_{\text{ob}}}\right)+\left(\frac{P_{r}^{M}+1-P_{r}^{C}}{P_{r}^{C}+1}\;\right). \end{array}$$

In the above equations, the condition CF_*s*+1_ and CF_*D*+1_ used to denote OB(PCI_*L*_, *P*_*r*_^*C*^) and OB(*S*_ob_, *P*_*r*_^*M*^ + 1) previous correlation, respectively. In this correlation process, the last concentration is provided if the constraint CF_*D*+1_ = CF_*s*+1_ + 1 (or) CF_*D*+1_ = CF_*S*_ob__ is verified. Therefore, the number of observation sessions in the above conditions retards the present session by augmenting the chances of precision in finding myocardial infarction. Hence, the present session observation in a different time interval is observed consecutively without additional analysis rate, diagnosis recommendation, and complexity. The previous two observations of OB∀ *S*_ob_ − 1 (or) PCI_*L*_ − 1 are again verified, and the session observation between the organization accumulate data based on *P*_*r*_ < *P*_*r*_^*M*^ + 1 and *P*_*r*_ < *P*_*r*_^*M*^. Case (i) analysis using the dataset information is presented in Table 1.

For the above observation data, the ECG observed is presented in Table 2.

The tabular analysis shows the common variation less observation for which CF_*S*_ observed is presented in Table 3. This observation is identified based on the above sequence, i.e., (1-4), (4-7), and (7-10). The learning process identifies *S* and *S* + 1 based on the mapping performed using *p*.

In Table 3, *p* in bold generates variations for the observations in different intervals. Therefore, the learning process identifies the above for CF_*D*_ such that its classification in (*D* + 1) or (*S* + 1) is analyzed. Based on this analysis, case (ii) classification is performed. In this case, the actual variation due to the concentrated values is identified with the different interval correlations. This is required for reducing the negative predictions in identifying PCI.

### 3.3. Case (ii) Analysis

In this case, the complexity and last known concentration due to prolonged assessment for (*S*_ob_ − *p*) are analyzed and observed based on different intervals. If this condition is not fairly addressed, then it outputs in precise session observation in high variations in blood flow and clot; hence, the successive value shift analysis is halted. The complexity of high blood pressure is identified in the condition *P*_*r*_^*M*^ + 1 obtaining different intervals to reduce the value shift check of *p* ∈ *S*_ob_. The remaining session observation has not been verified with the correlation and session observed. This myocardial infarction identification is verified with the help of value shift analysis and discussed in case (i) early detection of such infarction. Therefore, the analysis rate and complexity based on the condition *P*_*r*_^*M*^ < *P*_*r*_^*C*^ + 1 and  *P*_*r*_^*C*^ ≤ *P*_*r*_ are analyzed to ensure that the minimum satisfying condition of *P*_*r*_ = *P*_*r*_^*C*^ and *P*_*r*_ > *P*_*r*_^*C*^ is achieved. Based on the different intervals from the previous session observation, the value shift of OB(*S*_ob_, *P*_*r*_^*M*^ + 1) is along accounted for the two conditions as OB(PCI_*L*_, *P*_*r*_^*C*^) satisfied *P*_*r*_^*C*^ ≤ *P*_*r*_ and *P*_*r*_^*C*^ ≤ *P*_*r*_ ≤ *P*_*r*_^*M*^. The complexity in myocardial infarction identification outputs in normal heart functions and complexity in treating heart attack and cardiac arrest, and hence, the above cases (i) that fail CF are independently verified. The PCI value shift is observed and analyzed based on the heartbeat rate analysis of the deep learning in that knowledge gained from the previous observation. The above heart arrest identification indicates the failure condition of *P*_*r*_^*M*^ < *P*_*r*_^*C*^ + 1; then, output *P*_*r*_ > *P*_*r*_^*M*^ is nevertheless achieved. In Figure 4, the (*S* + 1) and (*D* + 1)-based learning process is illustrated.

In Figure 4, CF_*D*_ and CF_*S*_ are validated for (*S* + 1) and (*D* + 1) such that  *S* or *D* and shift outputs are observed. From the output, *D*, and shift with the correlating stored ECG data are analyzed for training. The proposed model verifies *P*_*r*_^*C*^ ≤ *P*_*r*_ until the heart arrest analysis based on the PCI level is identified, and diagnosis recommendation in different intervals is processed for value shift verification PCI_*L*_ ECG observation was provided alone. In this condition based on *P*_*r*_^*M*^ + 1 = *P*_*r*_^*M*^  and *P*_*r*_^*M*^ + 1 = *P*_*r*_ for validating the infarction rate. Therefore, the least possible condition of *P*_*r*_ ≤ *P*_*r*_^*C*^ is satisfied, and hence, the maximum session observation for achieving the condition CF_*S*_ob_−*p*_ and CF_*S*_ob_−*p*−1_ is (*C*)_*S*_ob_−*p*−1_ is retained with (1 − PCI_*L*_ + *S*_ob_ − 1)/*S*_ob_ and hence the value shift verification from identifying the myocardial infarction analysis in the different intervals for the real-time application services. Based on the above learning process, the shift occurred in different intervals for 10 observations are tabulated in Table 4.

In Table 4, the “bold” highlights refer to the normal observation whereas the rest represents the variations observed in the given time interval. Based on the above validation, the correlation between the normal ECG and concentrated values takes place. The varying ECG identifications based on the above shift values are presented in Table 5.

## 4. Discussion

Discussion presents the comparative analysis-based performance assessment of the proposed CVAM. The data from [29] is used for detecting abnormal and normal ECGs that cause myocardial infarction. This data source correlates 109446 samples under 125 Hz frequencies for categorizing 5 different observations. It contains 188 columns by observing ECG at different sessions and time intervals. For a common analysis, a maximum of 10 min observations is accounted for in this assessment. Based on this information, the sensitivity, specificity, precision, and negative prediction metrics are compared with ML-ResNet [23], TSCNN [27], and Big-ECG [17] techniques.

### 4.1. Sensitivity Comparison

In Figure 5, the variations in blood flow and clot are observed through previous correlation, and ECG monitoring identifies blockage of blood in the vessels; outputs in myocardial infarction are to improve the session observation, and normal data correlation through the PCI level does not provide complexity, and diagnosis recommendation depends on the training instance using deep learning based on heartbeat, blood pressure, and flow rate analysis in different time intervals. The learning paradigm trained based on the sessions and normal observation data condition *P*_*r*_ ∈ [*P*_*r*_^*M*^ + 1, *P*_*r*_^*C*^] and previous observation sessions from the initial ECG observation enhance the sensitivity and specificity and are analyzed for early diagnosis wherein the PCI value shift due to blocks based on such infarction detection can be observed. This negative prediction is addressed using deep learning, and the last known concentration can be observed for satisfying successive analysis based on the training and PCI level verification for myocardial infarction, preventing negative prediction. Therefore, the application value of remote ECG monitoring ensures complexity is reduced, preventing high sensitivity due to new session observation.

### 4.2. Specificity Comparison

The PCI level is recommended for the patients based on the session observation, and normal data correlation ensures diagnosis recommendation for detecting myocardial infarction analysis; the value shift due to blocks for the above factors with the ECG values as first input observation based on different variations in blood flow and clot is observed and analyzed for providing diagnosis recommendation to the patients based on the condition argmin ∑_*t*=1_^*V*_*i*_^(*P*_*r*_^*M*^)_*t*_∀ [*P*_*r*_^*M*^ − *P*_*r*_^*C*^], and session observation is represented in Figure 6. This proposed CVAM satisfies high sensitivity and specificity by estimating the normal heart function instances to the present variations in the blood vessels. In this observation, the ECG monitoring is observed for identifying cardiac arrest and heart arrest through deep learning until a new session observed based on PCI value shift at different time intervals, prevents the negative prediction, and identifies the myocardial infarction mitigation based on the ECG monitoring, and previous correlation is computed during training of the session and normal observation data. Therefore, the session observation and correlation through the learning process maximized specificity, and complexity based on variations in the blood flow is high specificity with diagnosis recommendation precision.

### 4.3. Precision Comparison

In this proposed session, observation and normal data correlation process achieves high precision and sensitivity depending on ECG monitoring, and previous correlations based on identifying acute myocardial infarction at different intervals of time are used for detecting the negative prediction (refer to Figure 7). The sequential process of ECG observations and different patient monitoring based on normal heart functions is alleviated and the PCI value shifts for observing the variations in the normal ECG values due to different heart rates. The cardiac arrest identification based on the normal heart function using the accumulated and organized infarction rate validation about the ECG value assessment based on deep learning in different intervals for validating sequential complexity in identifying myocardial infarction for reducing the negative predictions based on the variations in the blood flow enhances the precision and sensitivity in the early diagnosis of PCI during myocardial infarction detection. Therefore, the training based on session and normal observation data computation depend on other factors in the PCI based on ECG monitoring, and therefore, the precision is high, and diagnosis recommendation also increases.

### 4.4. Negative Prediction Comparison

This proposed model for monitoring and analyzing normal heart functions of the patients for identifying any changes in blood vessels at different time intervals and other factors based on session observation and normal data correlation does not provide acute myocardial infarction based on ECG monitoring and previous correlation. The computation of the training instance and diagnosis recommendation in the above analysis based on the deep learning and ECG values correlates for precisely determining PCI from the last known concentration based on the condition *P*_*r*_ ∈ [*P*_*r*_^*M*^ + 1, *P*_*r*_^*C*^]∀ (*p* + 1) estimated using infarction rate validation for the condition (PCI_*L*_ − *S*_ob_) relies on the balancing of sensitivity and specificity instances analyzed for the above condition of session observation. Based on the training instance, the cumulative sessions and PCI level-based infarction rate analysis with the session and normal observation data through deep learning prevent negative prediction. The proposed model provides acute myocardial infarction observation based on the normal heart function for which previous correlation achieves less negative prediction as presented in Figure 8. For the above metrics, the summary is presented in Tables 6 and 7 for observed sessions and shift factors.

## 5. Conclusion

In this article, a concentrated value assessment model is introduced for strengthening PCI treatment levels in diagnosing PCI. In this model, the ECG and its associated data from different observation sessions are used for identifying PCI. Specifically, the proposed model identifies the shift in ECG data over the continuous observation interval. The associated data is analyzed for its concentration and impact over the varying session intervals for identifying the PCI treatment level for the user/patient. The normal user data is correlated with the analyzed data for preventing negative predictions. In this correlation process, deep learning is employed for classifying variations based on ECG data shift and normal data. This process relies on variation shift-based training for which the accompanying data concentration is analyzed for preventing negative correlation outputs. Based on the session and errorless outputs, the learning model is consecutively trained for identifying the shifts in ECG data analysis. From the experimental analysis, it is seen that the proposed model achieves 7.4% high sensitivity, 7.93% specificity, 13.83% high precision, and 13.83% less negative prediction for the varying observed sessions.

## Figures and Tables

**Figure 1:** Proposed model.

**Figure 2:** *P*_*r*_^*C*^ and *S*_op_-based observation.

**Figure 3:** Learning—normal data correlation.

**Figure 4:** Learning—(*S* + 1) and (*D* + 1).

**Figure 5:** Sensitivity.

**Figure 6:** Specificity.

**Figure 7:** Precision.

**Figure 8:** Negative prediction.

**Table 1:** Observed data for normal and varying sessions.

Time (min)	1-2	2-3	3-4	4-5	5-6	6-7	7-8	8-9	9-10
Observation 1	1.00*E* + 00	7.58*E* − 01	1.12*E* − 01	0.00*E* + 00	8.06*E* − 02	7.85*E* − 02	6.61*E* − 02	4.96*E* − 02	4.75*E* − 02
Observation 2	9.08*E* − 01	7.84*E* − 01	5.31*E* − 01	3.63*E* − 01	3.66*E* − 01	3.44*E* − 01	3.33*E* − 01	3.08*E* − 01	2.97*E* − 01
Observation 3	7.30*E* − 01	2.12*E* − 01	0.00*E* + 00	1.19*E* − 01	1.02*E* − 01	1.02*E* − 01	1.11*E* − 01	1.24*E* − 01	1.15*E* − 01
Observation 4	1.00*E* + 00	9.10*E* − 01	6.81*E* − 01	4.73*E* − 01	2.29*E* − 01	6.88*E* − 02	0.00*E* + 00	4.17*E* − 03	1.46*E* − 02
⋮	⋮	⋮	⋮	⋮	⋮	⋮	⋮	⋮	⋮
Observation 10	1.00*E* + 00	9.14*E* − 01	4.74*E* − 01	0.00*E* + 00	6.43*E* − 02	3.18*E* − 01	4.05*E* − 01	3.92*E* − 01	3.82*E* − 01

**Table 2:** ECG observed.

Time (min)	1-4			4-7			7-10		
Observation 1									
Observation 2									
Observation 3									
Observation 4									
⋮	⋮	⋮	⋮	⋮	⋮	⋮	⋮	⋮	⋮
Observation 10									

**Table 3:** *S* and *S* + 1 for the above representation.

Time (min)	1-4			4-7			7-10		
	*S*	*S* + 1		*S*	*S* + 1		*S*	*S* + 1	
Observation 1	1.00*E* + 00	—		8.68*E* − 01	—		6.23*E* − 01		
Observation 2	9.54*E* − 01	—		8.87*E* − 01	—		6.82*E* − 01	6.65**E** − 01	
Observation 3	8.80*E* − 01	—		8.90*E* − 01	—		5.60*E* − 01		
Observation 4	9.10*E* − 01	**0.022138**		8.94*E* − 01	—		6.44*E* − 01	6.81**E** − 01	
⋮	⋮	⋮	⋮	⋮	⋮	⋮	⋮	⋮	⋮
Observation 10	8.42*E* − 01	—		9.05*E* − 01	—		6.68*E* − 01		

**Table 4:** Shift detection in different intervals.

Time (min)	1-4	4-7	7-10	1-4	4-7	7-10
	(*S* + 1)			(*D* + 1)		
Observation 1	**0**	0.032377	0.064753	**0**	0.045788	0.036098
Observation 2	0.064058	0.052827	0.126103	0.013317	0.079809	0.0269
Observation 3	0.013008	0.021301	0.190856	0.001981	**0**	**0**
Observation 4	0.051051	0.047964	0.303724	0.002986	0.214765	**0**
⋮	⋮	⋮	⋮	⋮	⋮	⋮
Observation 10	**0**	0.018644	0.303724	0.007494	0.045296	**0**

**Table 5:** ECG shift observation.

Time (min)	1-4	4-7	7-10	1-4	4-7	7-10
	(*S* + 1)			(*D* + 1)		
Observation 1	0			0		
Observation 2						
Observation 3					0	0
Observation 4						0
⋮	⋮	⋮	⋮	⋮	⋮	⋮
Observation 10	0					0

**Table 6:** Comparative analysis summary for observed sessions.

Metrics	ML-ResNet	TSCNN	Big-ECG	CVAM	Findings
Sensitivity	0.897	0.953	0.928	1	7.4% high
Specificity	0.794	0.826	0.904	1	7.93% high
Precision	0.582	0.692	0.815	0.973	13.83% high
Negative prediction	0.133	0.121	0.095	0.0673	9.81% less

**Table 7:** Comparative analysis summary for shift factor.

Metrics	ML-ResNet	TSCNN	Big-ECG	CVAM	Findings
Sensitivity	0.526	0.708	0.862	1	7.5% high
Specificity	0.383	0.615	0.768	1	8.23% high
Precision	0.57	0.696	0.816	0.951	12.85%high
Negative prediction	0.138	0.118	0.093	0.0631	10.65% less

## Data Availability

No data were used to support this study.

## References

[1] Kim M. G., Ko H., Pan S. B. (2020). A study on user recognition using 2D ECG based on ensemble of deep convolutional neural networks. *Journal of Ambient Intelligence & Humanized Computing*.

[2] Rateb A. M. (2020). A fast compressed sensing decoding technique for remote ECG monitoring systems. *IEEE Access*.

[3] Bu Y., Hassan M. F. U., Lai D. (2020). The embedding of flexible conductive silver-coated electrodes into ECG monitoring garment for minimizing motion artefacts. *IEEE Sensors Journal*.

[4] Schmitz T., Wein B., Methe H. (2022). Association between admission ECG changes and long-term mortality in patients with an incidental myocardial infarction: results from the KORA myocardial infarction registry. *European Journal of Internal Medicine*.

[5] Scally C., Choo W., Rudd A. (2020). The early dynamic of ECG in Takotsubo syndrome presenting with ST-elevation: a comparison with age and gender-matched ST-elevation myocardial infarction. *International Journal of Cardiology*.

[6] Yen K. C., Chan Y. H., Wu C. T. (2021). Resuscitation outcomes of a wireless ECG telemonitoring system for cardiovascular ward patients experiencing in-hospital cardiac arrest. *Journal of the Formosan Medical Association*.

[7] Taha Y., Bhatt D. L., Mukherjee D. (2020). Early post-percutaneous coronary intervention chest pain: a nationwide survey on interventional cardiologists' perspective. *Cardiovascular Revascularization Medicine*.

[8] Fakhri Y., Andersson H., Gregg R. E. (2021). Diagnostic performance of a new ECG algorithm for reducing false positive cases in patients suspected acute coronary syndrome. *Journal of Electrocardiology*.

[9] Zhang F., Wang J., Shao X. (2022). Longitudinal evaluation of diastolic dyssynchrony by SPECT gated myocardial perfusion imaging early after acute myocardial infarction and the relationship with left ventricular remodeling progression in a swine model. *Journal of Nuclear Cardiology*.

[10] Faramand Z., Frisch S. O., DeSantis A. (2019). Lack of significant coronary history and ECG misinterpretation are the strongest predictors of undertriage in prehospital chest pain. *Journal of Emergency Nursing*.

[11] Wang G., Zhao Q., Cheng Q., Zhang X., Tian L., Wu X. (2019). Comparison short time discharge with long time discharge following uncomplicated percutaneous coronary intervention for non-ST elevation myocardial infarction patients. *BMC Cardiovascular Disorders*.

[12] Wasimuddin M., Elleithy K., Abuzneid A. S., Faezipour M., Abuzaghleh O. (2020). Stages-based ECG signal analysis from traditional signal processing to machine learning approaches: a survey. *IEEE Access*.

[13] Liu X., Wang H., Li Z., Qin L. (2021). Deep learning in ECG diagnosis: a review. *Knowledge-Based Systems*.

[14] Kim J., Cho Y. S., Lee B. K. (2021). Diagnostic value of transthoracic echocardiography compared to electrocardiogram in predicting coronary artery stenosis among patients after cardiac arrest. *The American Journal of Emergency Medicine*.

[15] de Freitas Silva E., Cardinalli-Neto A., Grassi L. V., Nogueira P. R., Bestetti R. B. (2021). Noninvasive prediction of late potentials in the signal-averaged ECG in patients with chronic Chagas disease. *Journal of Electrocardiology*.

[16] Fu Y., Pan Y., Gao Y., Yang X., Chen M. (2021). Predictive value of CHA2DS2-VASc score combined with hs-CRP for new-onset atrial fibrillation in elderly patients with acute myocardial infarction. *BMC Cardiovascular Disorders*.

[17] Xu Y., Yu Y., He L., Wang Y., Gu Y. (2022). Predicting efficacy of combined assessment with fragmented QRS and severely depressed heart rate variability on outcome of patients with acute myocardial infarction. *Heart and Vessels*.

[18] Hussain I., Park S. J. (2021). Big-Ecg: cardiographic predictive cyber-physical system for stroke management. *IEEE Access*.

[19] Ko H., Pan S. B., Měsíček L. (2020). Personal identification study for touchable devices with ECG, concurrency and computation-practice & experience. *Concurrency and Computation: Practice and Experience*.

[20] Bigler M. R., Zimmermann P., Papadis A., Seiler C. (2021). Accuracy of intracoronary ECG parameters for myocardial ischemia detection. *Journal of Electrocardiology*.

[21] Hariharan S., Gupta M. (2020). Improving cloud-based ECG monitoring, detection and classification using GAN. *Fusion: Practice and Applications*.

[22] Jiao Y., Qi H., Wu J. (2022). Capsule network assisted electrocardiogram classification model for smart healthcare. *Biocybernetics and Biomedical Engineering*.

[23] Gupta S., Agnihotri S., Birla D., Jain A., Vaiyapuri T., Lamba P. S. (2021). Image caption generation and comprehensive comparison of image encoders. *Fusion: Practice and Applications*.

[24] Tadesse G. A., Javed H., Weldemariam K. (2021). DeepMI: deep multi-lead ECG fusion for identifying myocardial infarction and its occurrence-time. *Artificial Intelligence in Medicine*.

[25] Zhao Y., Xiong J., Hou Y. (2020). Early detection of ST-segment elevated myocardial infarction by artificial intelligence with 12-lead electrocardiogram. *International Journal of Cardiology*.

[26] Zhang Y., Sun L., Song H., Cao X. (2014). Ubiquitous WSN for healthcare: recent advances and future prospects. *in IEEE Internet of Things Journal*.

[27] Fatimah B., Singh P., Singhal A., Pramanick D., Pranav S., Pachori R. B. (2021). Efficient detection of myocardial infarction from single lead ECG signal. *Biomedical Signal Processing and Control*.

[28] Elngar A. A., Arafa M., Fathy A. (2021). Image classification based on CNN: a survey. *Journal of Cybersecurity and Information Management*.

[29] Han C., Shi L. (2020). ML–ResNet: a novel network to detect and locate myocardial infarction using 12 leads ECG. *Computer Methods and Programs in Biomedicine*.

[30] Li W., Tang Y. M., Yu K. M., To S (2022). SLC-GAN: an automated myocardial infarction detection model based on generative adversarial networks and convolutional neural networks with single-lead electrocardiogram synthesis. *Information Sciences*.

[31] Aldana Blanco A. L., Grautoff S., Hermann T. (2020). ECG sonification to support the diagnosis and monitoring of myocardial infarction. *Journal on Multimodal User Interfaces*.

[32] Thorén A., Rawshani A., Herlitz J. (2020). ECG-monitoring of in-hospital cardiac arrest and factors associated with survival. *Resuscitation*.

